The article "Protection and Planning of Historic Districts Based on Internet of Things Perception" was published in 2022. Journal: Comput Intell Neurosci.

# Protection and Planning of Historic Districts Based on Internet of Things Perception

**DOI:** 10.1155/2022/1325381

**Published:** 2022-06-09

**Authors:** Qing Zhao, YunYing Ren

**Affiliations:** ^1^College of Urban and Environmental Sciences, Northwest University, Xi'an 710000, China; ^2^Architecture College, Xi'an University of Architecture and Technology, Xi'an 710000, China

## Abstract

With the development of the Internet of Things era, the Internet of Things technology has been gradually accepted by people and gradually entered the category of block management, but the specific practical application scope is not wide enough. At present, the community management of residents in blocks generally adopts closed management, and there are some problems such as insufficient scope of property management, weak strength, and serious waste of human resources. Incomplete development of the hidden value is of cultural tourism blocks. At the same time, there are still some problems in the traffic management of blocks, such as incomplete monitoring scope and weak supervision. Therefore, this study proposes a bilevel programming model to solve the optimization scheme of block road network, adopts the complete information game model to analyze the imbalance between property and residents, and adopts the AHP fuzzy evaluation method to detect the current life happiness coefficient of urban residents and collect residents' suggestions for the future planning of historical blocks. Because the perception layer of the Internet of Things has the advantages of rapidity, accuracy, and unmanned operation, it can contribute a practical force to the protection and planning of historical blocks quickly and at low cost.

## 1. Introduction

In urban block planning, there are some problems in China, such as community closed pipe, crowded traffic routes, insufficient utilization of infrastructure, and so on [1]. However, in the era of big data information explosion in 2022, the digital information of urban blocks is bound to be on the right track, so the ancient survival mode of urban blocks has to lead to new changes. However, for some cities, some blocks have famous places of interest or rare regional characteristics, which is a pity to be destroyed. It is better to adopt Kevin Lynch's point of view that by protecting ancient buildings, we are preserving a sense of honor and history [2]. Therefore, the application of Internet of Things technology to the protection and planning of historical blocks has become the theme of urban planning in the new era.

The current situation of unreasonable infrastructure planning is the fatal factor of urban planning problems in developing countries in the world [3]. The infrastructure system of the neighborhood has a long service life, and the impact on the environmental conditions lasts for a long time. Therefore, the strategic planning process of block facilities helps to realize the vision of environmental sustainability. Long-term investment in potentially destructive facilities may mean that sustainability priority principles are not included in planning and construction projects because these projects often follow the old planning model.

In the protection and planning of historical blocks, the first thing that should be built and improved is the community management mode. As early as 2000, China defined the community as the community of people's social life within a certain geographical scope for the first time in the article “Opinions of the Ministry of Civil Affairs on Promoting Urban Community Construction in China” [4]. Since then, the community has been formally determined as a unit of urban development. At present, our community is basically closed, and the happiness coefficient of people's life is low, so we need to make reasonable planning and build the community into an open one. Starting from the perception layer of Internet of Things, this study explores the imbalance between property and residents by using the game model [5]. Second, AHP fuzzy evaluation is used to detect the current life happiness coefficient of urban residents and collect the focus of residents on community reform [6].

Second, we should study the rational development of cultural blocks on the premise of protection under the new technology. At present, China has tried to apply the Internet of Things technology to some historical and cultural blocks, but it is in an embarrassing situation that the application technology is not mature enough and the scope is not comprehensive enough. These blocks mainly take tourism industry as the development economy, and the activities of tourists from all over the world in this area have become one of the main sources of economic income for local cultural blocks. Therefore, in order to ensure the continuous input of sufficient passenger flow, we can design an intelligent bus system with the traffic demand of tourists as the guide [7]. At the same time, it is necessary to make reasonable planning for the allocation of cultural blocks in order to seek the result of maximizing the use of value [8].

Finally, with the technical support of the Internet of Things, the optimized road network of urban block traffic routes is designed. Simon, an outstanding scholar, put forward the concept of “satisfaction criterion,” which defines that people are more inclined to make decisions that best meet their own needs, rather than theoretically optimal decisions [9]. Sun Yan designed a route selection model for passengers under the dual influence of rationality and preference [10]. Liu Kai designed a route selection model including three aspects: selection habits, traffic information, and time prediction [11]; Xu Hongli designed a path selection model for road risk avoidance and inertia decision [12]. Based on the achievements of the above scholars, this study puts forward a bilevel programming model to explore the optimization scheme of network route [13].

## 2. Protection and Planning of Residential Communities

Under the transformation of the Internet of Things perception technology, the future of residential communities is bound to be based on openness. The mobility of people in the community is strengthened, the freedom of residents' living activities is wider, and the work of people in all aspects of the property will be more flexible and meticulous. Community functions, including community population management, community business management, community sports management, community security management, and other management modules, will be improved accordingly, so as to seek the simultaneous improvement of residents' freedom of activities and happiness coefficient.

### 2.1. Research on Property Management under the Game Theory Model

After the opening of the block, the number of people and vehicles in the community increased, which had an impact on the living comfort and the overall environment of the community, and the pressure on the property management department increased sharply. Therefore, it is necessary for the Internet of Things to fully coordinate the relationship among property management departments, community owners, and outsiders in the community. Among these three relationships, the property management department as the middle coordinator, its position is particularly important, so is the introduction of game theory knowledge to analyze the sustainable development of property management after the block opening.

In the analysis, we can know that both property enterprises and owners are rational economic people. Therefore, in community management, property managers and owners are principals and agents, respectively, so we can use the complete information game model to analyze the imbalance between owners and properties [14].

#### 2.1.1. Model Assumptions

The research objects of the model are residents and property companies.

The strategy of the game model: assuming that the owner of the game party is *N*1, the strategy adopted by the owner is as follows: one is to pay the property fee regularly, which makes the property company gain profits and have the motivation to continue management, and the other is not to pay the property fee on time, so *N*1 = (pay the property fee on time, not pay the property fee on time). The property of the other parties participating in the game is *N*2, which can get property fees on time by actively providing services, but cannot collect property fees on time by passively providing services, that is, *N*2 = (high-quality services, low-quality services).

#### 2.1.2. Modelling

Assuming that the income obtained by the property company under normal operation is *M* and the extra income obtained by the property fee collected by the property company is *E*, if the cost incurred by the property company in providing high-quality services for the owners is *C*1 and if the services provided by the property company are low cost, then the cost incurred by the property company at this time is *C*2, and at this time, *C*1 > *C*2.

When the property company provides high-quality services, such as good control of foreigners, timely provision of on-site warranty services, and property safety of owners, the community residents will generate income and assume *R*1. When the property company provides negative business services to residents, the income generated by residents is *R*2. Once residents refuse to pay property fees on the grounds of poor service of property companies, the amount will be used for residents' consumption of other matters, and the resulting income will be *E*. In terms of residents' income, the income of residents enjoying high-quality services must be greater than that of receiving low-quality services, that is, *R*1 > *R*2.

In this asymmetric nonzero game, no matter whether the property company provides quality management work or not, it will first consider delaying the payment of property fees. At this time, the income of residents is *R* or *R*2+*E*2. Property companies usually adopt the negative service mode, that is, *M*+*E*1 − *C*2, as given in Table 1.

#### 2.1.3. Model Solving

Let *α*(0 < *α* < 1) be the discount factor between residents and properties. If residents fail to pay fees on schedule, the benefits obtained by the owners are *R*1+*E*2, not the income of the unit *R*1. The owner's deferred payment behavior will lead to the inability of the property to provide high-level property management work, and the owner can get the benefit of *R*2+*E*2. Residents choose to pay on time according to the service quality of the property and should meet the following conditions:

(1) $$\begin{array}{c} \left(R1+E2\right)+\alpha \left(R2+E2\right)+\alpha 2\left(R2+E2\right)+\cdots \leq R1+\alpha \;R1+\alpha 2R1+\cdots ,\\ \text{Available after transformation }\left(R1+E2\right)+\frac{\alpha \left(R2+E2\right)}{1-\alpha }\leq \frac{R1}{1-\alpha }. \end{array}$$

When *α* ≥ *E*2/*R*1 − *R*2 appears, it indicates that the community property provides high-quality services, so the owner will not take the initiative to delay payment.

As for that behavior of property company, if the property company chooses nonquality service when serving the owner, at this stage, the benefit that the property management company can get is *M*+*E*1 − *C*2, not *M*+*E*1 − *C*1. The behavior of the property management company will cause the owner to delay payment, which makes the income of the property management company M-C2 in each stage. If the owner can pay on time, the property management company will not adopt the strategy of low-quality service. It can be expressed as follows [15]:

(2) $$\begin{array}{c} \left(M+E1-C2\right)+\alpha \left(M-C2\right)+\alpha 2\left(E-C\right)+\cdots \leq \left(M+E1-C1\right)+\alpha \left(M+E1-C1\right)+\cdots , \end{array}$$

i.e.,

(3) $$\begin{array}{c} \left(M+E1-C2\right)+\frac{\left(M-C2\right)\alpha }{1-\alpha }\leq \frac{M+E2-C1}{1-\alpha }. \end{array}$$

Solution is as follows:

(4) $$\begin{array}{c} \alpha \geq \frac{C1-C2}{E1}. \end{array}$$

When *α* ≥ *C*1 − *C*2/*E*1, residents pay property fees on time, and property companies provide high-quality services for residents.

According to the knowledge of game theory, if the number of times of the same result in the experiment reaches a certain value, then the payment vector can be obtained by a subgame equilibrium. In property management, if *α* can satisfy *α* ≥ *E*2/*R*1 − *R*2 and *α* ≥ *C*1 − *C*2/*E*1, the trigger strategy is a subgame equilibrium of infinite repeated game, while the service management of property and the on-time payment of residents are the equilibrium results of each stage, in which *α* represents the patience or concern of participants in property management.

### 2.2. Residents' Satisfaction under AHP Fuzzy Evaluation

At present, community construction services are mainly concentrated in three aspects: social welfare services for vulnerable groups, collective routine services, and convenient services [16].

When the community becomes open, the flow of foreign personnel and vehicles continues to increase. The safety risk factors are gradually improved. At the same time, property management immediately changed from closed management service to open service. During this period, there will inevitably be inadaptability and neglect of work, so the corresponding service quality provided by the property to residents will also be impacted. Therefore, it is of great practical significance for the future planning of the block to design a scientific evaluation model based on the perception layer technology of the Internet of Things and explore the true inner thoughts of residents.

#### 2.2.1. AHP Principle of Index Selection for the Evaluation Model

1. People-oriented principle: we should take the residents' own interests as the core of all works and fully meet the material and spiritual needs of residents [17].
2. The scientific nature of the evaluation index: it is the inevitable requirement of scientific and effective research results that we carry out rational screening on various needs of residents through comparative experiments and comparisons.
3. Systematicness of evaluation index: community management includes many aspects such as environmental safety, pension, residents' health, basic medical care, and convenient service. Therefore, these factors should be fully considered in the setting process of the evaluation system, so as to make the evaluation system holistic.
4. Principle of regional differences [18]: the design of the evaluation system should fully consider the different needs of different regions, For example, some communities where older people live should consider community healthcare and community medical care, while white-collar communities may pay more attention to community health and community entertainment and should consider the impact of outsiders on a series of public infrastructure enjoyed by the community after the implementation of the block system.

#### 2.2.2. AHP Index Weight of the Evaluation Model

This model is divided into first-class weights and second-class weights, with 6 first-class weights and 11 second-class weights. The first-level weight security includes two second-level weights, community security and personal and property safety, convenience includes the convenience of residents' lives and the speed of solving residents' difficulties, reliability includes property to residents' living guarantee and property to residents' safety guarantee, rapidity includes property companies' service speed and property companies' difficulty solving speed, economy mainly refers to residents' payment ratio, and comfort includes owners' living environment and owners' living happiness. Because the AHP evaluation model reflects the satisfaction index of community residents for the quality of property services as a whole, rather than an individual satisfaction index, it is necessary to avoid individual economic differences of residents. Using the proportion of payment as the second-class weight is an effective index to reflect the overall satisfaction of residents, so it is feasible. Each weight relationship is shown in Figure 1.

#### 2.2.3. Experimental Simulation of the AHP Evaluation Model

(1) Establish a hierarchical structure model: the index weight is set as target layer A, the first-level weight is criterion layer B, and the second-level weight is index layer C.

(2) Constructing judgment matrix: we compare several indicators at the same level that affect the satisfaction of owners with the construction of smart communities and compare the influence degree of the indicators at the upper level in pairs, thus forming a judgment matrix. After that, each index of the same layer is compared with the corresponding index of the previous layer in pairs, and finally, the relative importance of each factor of each layer is judged, respectively.

(3) Single arrangement of layers and total arrangement of layers: in this study, well-known property companies in Qingdao, such as New Age Property and Yinshengtai Property, are selected, and senior representatives of some community owners' committees are recruited to form an evaluation team to evaluate the index evaluation system of smart communities. Through in-depth interviews, the importance of each factor at the criterion level and index level is scored by the scaling method [19]. The specific scores obtained are given in Table 2.

Taking “security” as an example, the judgment matrix is constructed as *B*_1_:

(5) $$\begin{array}{c} B_{1}=\left[\begin{array}{ccc} 1 & \frac{1}{5} & \frac{1}{9}\\ 5 & 1 & \frac{1}{3}\\ 9 & 3 & 1 \end{array}\right]. \end{array}$$

In the **B**_1_ matrix, the index relationship represented by each data is as follows: **A**_12_=1/5: “Community security” is more important than “resident's property security.” **A**_13_=1/9: the importance of “personal safety of residents” is far greater than that of “property safety of residents.” **A**_23_=1/3: “Community security work” is slightly more important than “property safety of owners.”

(4) Consistency test of matrices: the steps of calculation by the summation method are as follows:

**Step 1 .**

Normalize the elements of *B* by column [20].

**Step 2 .**

$\bar{B}=\left(\bar{B\text{ij}}\right),\bar{B\text{ij}}=bij/\sum_{i=1}^{n}b_{ij},i,j=1,2,L,L,n.$

**Step 3 .**

Add $\bar{B}$ by rows to get $\bar{F}=\left[\bar{f1},\bar{f2}L\;L\;\bar{fn}\right],\bar{fi}=\sum \begin{array}{c} n\\ i=1 \end{array}bij$.

**Step 4 .**

After normalization $\bar{F}$, get $F=\left[\bar{f1},\bar{f2}L\;L\;\bar{fn}\right]T,K1=\bar{K}i/\sum_{i=1}^{n}{\bar{K}}_{i}$.

Table 3 provides the judgment matrix, results, and *fi* results of safety in the evaluation of residents' satisfaction with development community construction.

There is *aij*=*aik*/*akj*(*k*=1,2,…, *n*) for any *i*, *j*=1,2,…, *n*. When the matrices are completely consistent, there is *λ*_max_=*n*; when there is consistency error in the judgment matrix, *λ*_max_ > *n*. At the same time, the greater the error, the greater the value of *λ*_max_.

(6) $$\begin{array}{c} \lambda_{\max}=\frac{1}{n}\sum_{i=1}^{n}\frac{\sum_{j=1}^{n}a_{ij}k_{j}}{k_{j}}. \end{array}$$

The *λ*_max_ value of the judgment matrix of residents on the safety index of the development community is 3.1384.

C.I is used as an index to test the consistency of the above judgment matrix:

(7) $$\begin{array}{c} C.I=\frac{\lambda_{\max}-n}{n-1}=0.0135. \end{array}$$

After calculation, when *n* = 3, the correction coefficient R.I = 0.49.

Therefore, there is *C*.*R*=*C*.*I*/*RI*=0.0135/0.49=0.027551 < 0.1, so it is concluded that the judgment matrix is consistent. In the same way, the values of other weights can be calculated.

When the judgment matrix of “convenience **B**_2_” is $B_{2}=\left[\begin{array}{ccc} 1 & 5 & 9\\ 5 & 1 & 4\\ 1/9 & 1/4 & 1 \end{array}\right]$, the weight vector *F*_2_={0.7241, 0.1883}. When the judgment matrix of “reliability **B**_3_” is $B_{3}=\left[\begin{array}{cccc} 1 & 1/5 & 1/9 & 1/3\\ 5 & 1 & 1/3 & 3\\ 9 & 3 & 1 & 6\\ 3 & 1/3 & 1/6 & 1 \end{array}\right]$, the weight vector *F*_3_={0.2374, 0.4879}. When the judgment matrix of “rapidity **B**_4_” is $B_{4}=\left[\begin{array}{cc} 1 & 3\\ 1/3 & 1 \end{array}\right]$, the weight vector *F*_4_={0.2374, 0.4879}. When the judgment matrix of “Economy **B**_5_” is $B_{5}=\left[\begin{array}{ccc} 1 & 1/3 & 5\\ 3 & 1 & 7\\ 1/5 & 1/7 & 1 \end{array}\right]$, the weight vector *F*_5_={0.113, 0.2713}. When the judgment matrix of “Comfort Β6” is $B6=\left[\begin{array}{ccc} 1 & 4 & 8\\ 1/4 & 1 & 7\\ 1/8 & 1/8 & 1 \end{array}\right]$, the weight vector *F*6={0.5328, 0.0654, 0.635, 0.3112}.

By the same token, the judgment matrix of the first-level index **B** in the AHP evaluation model is

(8) $$\begin{array}{c} B=\left[\begin{array}{cccccc} 1 & 0.1358 & \frac{1}{2} & \frac{1}{5} & 0.11 & \frac{1}{3}\\ 6 & 1 & 6 & 2 & \frac{1}{3} & 3\\ 2 & 0.2321 & 1 & 0.2 & 0.2321 & 0.2\\ 1 & 4 & 5 & 1 & \frac{1}{5} & 3\\ \frac{1}{4} & 1 & 7 & 5 & 1 & 5\\ 3 & \frac{1}{4} & 5 & \frac{1}{3} & \frac{1}{5} & 1 \end{array}\right],\\ F=\left\{0.0283,0.2496,0.0325,0.4289,0.0831\right\}. \end{array}$$

From this, the values of the weights of each level of the final evaluation model can be obtained, as given in Table 4.

#### 2.2.4. Experimental Conclusions of the AHP Evaluation Model

From the AHP evaluation model, we can see that in the future open community planning, the security and convenience of the community are extremely important. First of all, the safety management of the community should be strengthened, but more cameras must be placed to check suspicious things, so as to ensure that there is no dead angle in the photography field of vision and achieve the effect that the security system can effectively meet the development needs. Second, a set of risk prevention measures should be scientifically formulated to avoid the occurrence of sudden dangerous events.

Due to the serious aging trend in today's society, the proportion of children and children is increasing, and the services for the life, health, and personal safety of the elderly and children are also extremely important, so the community residents' service health platform should be added. It can provide physical examination services or medical services for a certain period of time and can also install some health monitoring instruments, such as the pulse test, blood sugar test, and body fat measurement, and can provide residents with physical fitness tests free of charge at any time.

In the future block planning work, in the community construction module, we should first meet the needs of residents and take the residents' true happiness experience as the core essence. From the community life, environment, and other aspects of transformation, earnestly do a good job in the basic maintenance and transformation of the community.

## 3. Protection and Planning of Cultural Tourism Blocks

At present, the commercialization of historical sites is gradually becoming a status quo. Among them, most famous cultural blocks take tourist flow and tourist activity track as one of the main local economic sources. This situation makes the original sense of history greatly reduced, but the commercial money atmosphere is getting hotter and hotter, destroying the original antique cultural atmosphere. Therefore, we need to use the emerging Internet of Things technology to plan cultural tourism blocks on the premise of protection.

### 3.1. Problems

First of all, regional culture and commercialization are mixed. In cultural areas, all kinds of goods are sold, either in the form of stalls or in the form of shops set up with blocks as the background. Moreover, its products are various and mixed, and at the same time, the products have the attribute of gorgeous and bright colors, which easily causes tourists' aesthetic fatigue under the interweaving of various colors, thus leading to tourists' visual deviation of ancient buildings [21]. At the same time, vendors' cries are loud and messy, which will greatly damage the cultural atmosphere of the block.

Second, the demand for goods with cultural characteristics is not high. In the commercial area, catering and local specialties have become the hottest economic industries, while the goods related to local culture are widely sold on major network platforms, which makes them lose the tourism demand that they must buy in their areas, thus leading to the serious situation that the commercialization model is biased in some aspects.

### 3.2. Solution

First of all, functional zoning is carried out, which divides the cultural area from the commercial area, and at the same time, it is subdivided according to the types of goods sold. Second, the Internet of Things technology is implanted, and the Internet of Things is used to promote the mutual communication between various business styles in culture, so as to achieve the purpose of common progress. It can also realize the tripartite interaction among cultural products, tourists, and businesses, thus effectively realizing the reuse of cultural carriers and realizing the revolatilization of cultural functions in the process of cultural blocks. You can also use the Internet to build the connection with equipment and machines. For example, when the sensor detects that the decibel value is too high, it automatically sends information to each automatic noise reduction system. The system automatically identifies the noise area and turns on the noise reduction function at a special fixed point. The general flowchart of the idea is shown in Figure 2.

## 4. Optimization of the 3-Block Road Network

When residents face travel demand, they will have a variety of routes to choose. At the same time, the economic benefits and cost losses of each route are different, such as the environmental pollution value caused by vehicle exhaust, the consumption cost of vehicles, and the time value spent. Therefore, the method of using Internet of Things technology to study a route with low cost and high economic benefits is considerable.

### 4.1. Residents' Travel Route Choice Behavior

With the development of modern intelligent transportation technology based on Internet of Things technology, travelers can obtain the driving cost of *n* routes between starting and ending points through navigation tools (such as Baidu map, Tencent map, and Gaode map) and choose the route with lower cost according to preferences (shortest distance, shortest free flow time, and decision inertia). Before the opening of the closed block, because of its large size, urban travelers have a long detour distance, which is easy to produce the phenomenon of traffic superposition near it. After the block is opened, the roads inside the block will be made public, and travelers will have more choices, thus relieving the flow pressure of traffic roads in the surrounding areas. However, when urban travelers enter the block, they may face pedestrians crossing the street and motor vehicles stopping at the roadside. Therefore, when the difference between the travel cost across the block and the travel cost without crossing the block is within its acceptable range, travelers often refuse to choose the travel route across the block, that is, there is travel inertia.

### 4.2. Building a Bilevel Programming Model

#### 4.2.1. Lower Model

The travel route of residents in the block will definitely cross the block. If the flow of internal travelers on a certain path is positive, the travel cost of this path is less than that of other unused paths crossing blocks, and its complementary conditions can be expressed as

(9) $$\begin{array}{c} f_{ri,mi}^{w}\;\cdot \;\left(C_{ri}^{w}-\mu_{i}^{w}\right)=0,C_{ri}^{w}-\mu_{i}^{w}\geq 0,\;\forall ri\in R_{i}^{w},w\in W. \end{array}$$

where *mi* means the residents of the block, *f*_*ri*,*mi*_^*w*^ is the flow of travelers inside *ri* on the path across blocks, *C*_*ri*_^*w*^ is the travel cost of path *ri*, *μ*_*i*_^*w*^ is the minimum travel cost of crossing blocks between the OD pair *w*, and *R*_*i*_^*w*^ is the set of paths across blocks between OD pairs *w*.

For urban travelers, if the flow of urban travelers on a route aa crossing a block is positive, the travel cost of this route is less than that of other unused routes, and the complementary conditions are as follows:

(10) $$\begin{array}{c} f_{ri,m0}^{w}\;\cdot \;\left(C_{ri}^{w}-\mu_{r}^{w}\right)=0,C_{ri}^{w}-\mu_{r}^{w}\geq 0,\forall ri\in R_{i}^{w},\;\forall r\in R^{w},w\in W, \end{array}$$

where *m*0 means the city travelers, *f*_*ri*,*m*0_^*w*^ is the traffic of urban travelers on the path *ri*, *μ*_*r*_^*w*^ is the optimal travel cost between OD and *w*, *R*^*w*^ Ff is the set of all paths between OD pairs *w*.

If the flow of urban travelers on a path *r*0 that does not cross the block is positive, then for the urban travelers on the path, the travel cost of the path is less than the travel cost of other unused paths *ri* that do not cross the block, and the difference between the travel cost and the path within the block is less than the acceptable threshold *ε*_*w*_ of the travelers who choose the path, which can be expressed as

(11) $$\begin{array}{c} C_{r_{0}}^{w}-\mu_{0}^{w}\geq 0C_{r_{0}}^{w}\mu_{i}^{w}\geq \varepsilon_{w},\\ \text{if }f_{r_{0},m_{0}}^{w}=0,\;\forall r_{0}\in R_{0}^{w},\;\forall r_{i}\in R_{i}^{w},w\in W. \end{array}$$

(12) $$\begin{array}{c} C_{r_{0}}^{w}-\mu_{0}^{w}\geq 0C_{r_{0}}^{w}\mu_{i}^{w}\geq \varepsilon_{w},\\ \text{if }f_{r_{0},m_{0}}^{w}=0,\;\forall r_{0}\in R_{0}^{w},\;\forall r_{i}\in R_{i}^{w},w\in W, \end{array}$$

where *f*_*r*_0_,*m*_0__^*w*^ is the flow of urban travelers on the path *r*_0_, *C*_*r*_0__^*w*^ is the travel cost of path *r*_0_, *μ*_0_^*w*^ is the minimum travel cost between the OD pair *w* that does not cross the block, *R*_0_^*w*^ is the set of paths between OD pairs *w* that do not cross super blocks.

Formulas (11) and (12) are expressed as complementary conditions, and the transfer function is introduced [22]:

(13) $$\begin{array}{c} \gamma_{1}\left(\psi ,Г,\Lambda \right)=\left\{\begin{array}{cc} 0, & \text{if }\psi =0\;\&\&\;0\leq Г\leq \Lambda ,\\ \psi +Г, & \text{other}, \end{array}\right. \end{array}$$

where *ψ*, *Г*, Λ is an independent waste negative variable, which can be expressed in the following complementary form based on equations (11), (12), and (14):

(14) $$\begin{array}{c} f_{ri,m0}^{w}\;\cdot \;\left[\gamma_{1}\left(C_{r_{0}}^{w}-\mu_{0}^{w},C_{r_{0}}^{w}-\mu_{i}^{w},\varepsilon_{w}\right)\right]=0, \end{array}$$

where *γ*_1_(*C*_*r*_0__^*w*^ − *μ*_0_^*w*^, *C*_*r*_0__^*w*^ − *μ*_i_^*w*^,*ε*_*w*_) ≥ 0,  ∀ *r*_*i*_ ∈ *R*_0_^*w*^, *w* ∈ *W*.

The above complementary conditions (9), (10), and (14) can be extended to a mixed equilibrium model, which is expressed by the following mathematical programming model:

(15) $$\begin{array}{c} \min F=\left(f_{r_{i},m_{i}}^{w},f_{r_{i},m_{o}}^{w},f_{r_{o},m_{o}}^{w},\varepsilon_{w}\right)=\sum_{w\in W}\sum_{r_{i}\in R_{i}^{w}}f_{r_{i},m_{i}}^{w}\cdot \left(C_{r_{i}}^{w}-\mu_{r}^{w}\right)+\sum_{w\in W}\sum_{r_{i}\in R_{i}^{w}}f_{r_{i},m_{o}}^{w}\cdot \left(C_{r_{i}}^{w}-\mu_{r}^{w}\right)+\sum_{w\in W}\sum_{r_{o}\in R_{o}^{w}}f_{r_{o},m_{o}}^{w}\cdot \left[\gamma_{1}\left(C_{r_{0}}^{w}-\mu_{0}^{w},C_{r_{0}}^{w}-\mu_{i}^{w},\varepsilon_{w}\right)\right],\\ \sum_{w\in W}\sum_{r_{i}\in R_{i}^{w}}\delta_{r_{i},a}^{w}\cdot f_{r_{i},m_{i}}^{w}+\sum_{w\in W}\sum_{r_{i}\in R_{i}^{w}}\delta_{r_{i},a}^{w}\cdot f_{r_{i},m_{o}}^{w}+\sum_{w\in W}\sum_{r_{o}\in R_{o}^{w}}\delta_{r_{o},a}^{w}\cdot f_{r_{o},m_{o}}^{w}=x_{a},\;\forall a\in A,\\ \sum_{r_{i}\in R_{i}^{w}}f_{r_{i},m_{i}}^{w}+\sum_{r_{i}\in R_{i}^{w}}f_{r_{i},m_{o}}^{w}+\sum_{r_{o}\in R_{o}^{w}}f_{r_{o},m_{o}}^{w}=d_{m_{i}}^{w}+d_{m_{o}}^{w}\cdot \sum_{r_{i}\in R_{i}^{w}}P_{r_{i},m_{o}}+d_{m_{o}}^{w}\cdot \sum_{r_{o}\in R_{o}^{w}}f_{r_{o},m_{o}}=d_{w},\\ P_{r_{i},m_{o}}=P\left\{r_{i}|C_{k_{o}}^{w}-C_{r_{i}}^{w}\geq \varepsilon^{w}\right\}+P\left\{r_{i}|C_{k_{o}}^{w}-C_{r_{i}}^{w}\leq \varepsilon^{w}\right\}\cdot \tau ,\;\forall k_{o}\in K_{o},r_{i}\in R_{i},\\ P_{r_{i},m_{o}}=P\left\{r_{o}|C_{r_{o}}^{w}-C_{r}^{w}\leq 0\right\}+P\left\{r_{i}|C_{r_{o}}^{w}-C_{k_{i}}^{w}\leq \varepsilon^{w}\right\}\cdot \left(1-\tau \right),\;\forall r_{o}\in R_{o},\forall k_{i}\in R_{i},r\in R,\\ C_{r_{i}}^{w}-\mu_{i}^{w}\geq 0,\;\forall k_{i}\in R_{i}^{w},w\in W,\\ C_{r_{i}}^{w}-\mu_{i}^{w}\geq 0,\forall k_{i}\in R_{i}^{w},\;\forall r\in R^{w},w\in W,\\ \gamma_{1}\left(C_{r_{0}}^{w}-\mu_{0}^{w},C_{r_{0}}^{w}-\mu_{i}^{w},\varepsilon_{w}\right)\geq 0,\;\forall r_{i}\in R_{i}^{w},\forall r_{o}\in R_{o}^{w},w\in W. \end{array}$$

In the model, F represents the optimization function, which is used to obtain the overall minimum distance between block resident travelers and city travelers under complementary conditions (9), (10), and (14), that is, the sum of the distance between block resident travelers and equilibrium points and the distance between city travelers and equilibrium points is minimum.

#### 4.2.2. Upper Layer Model

In order to ensure that the optimized route of the block road network is more in line with the actual needs, this study constructs a planning model with the minimum total cost of the system under the conditions of multiple factors (travel cost, environmental factors, and potential safety hazards) as follows.

(1) Optimize the objective function: ignoring other factors, it is approximately considered that the travel cost is equal to the sum of the travel time cost and the travel cost itself, and the calculation formula is as follows [23]:

(16) $$\begin{array}{c} \min Tc=\left(\lambda \;\cdot \sum_{a0\in A0}ta0\;\cdot \;xa0+\sum_{a0\in A0}la0\cdot xa0\cdot ba0\right)+\left(\lambda \cdot \sum_{ai\in Ai}tai\cdot xaii+\sum_{ai\in Ai}tai\;\cdot \;xaii\cdot bai\right), \end{array}$$

where *Tc* is the total cost of road network driving, *λ* is the traveler's time value (VOT) parameter, *ta*0 and *tai* are the vehicle travel times of road sections *a*0 and *ai*, *la*0 and *lai* are the length of road sections, *xa*0 and *xai* are the road section flows, *ba*0 and *bai* are the unit operating expenses of cars, *A*0 is the collection of road sections outside the block, and *Ai* is the collection of sections within the block.

When the block is opened, the vehicle circulation inside it is more frequent, but the exhaust pollution emitted by a large number of vehicles during driving will seriously affect the residents and their surrounding environment. Therefore, when making decisions, it is necessary to bring the environmental pollution loss in the block into the optimization goal. The specific calculation formula is as follows:

(17) $$\begin{array}{c} \min Ec=\sum_{a0\in A0}Eai\cdot Qc, \end{array}$$

where *Ec* is the cost of environmental pollution loss, *Qc* is the average loss cost per unit pollutant (including tail gas treatment cost and health loss cost), and *Qc* is the unit road pollutant emissions; this study focuses on the calculation of the main pollutants (CO, HC, and NOX) produced when the vehicle exhaust emissions. The specific calculation formula is as follows [24]:

(18) $$\begin{array}{c} Eai=\sum_{k\in K}EFk\cdot xailai, \end{array}$$

where *EFk* is the emission factor of pollutant *k*, and *EFco*=0.5216*γco*, *EFHC*=0.0634*γHC*, *EFNOx*=0.0198*γNOx*, and *γCO*, *γHC*, and *γHC* are calculated as the velocity correction factors, which can be obtained from Table 5.

Existing studies have shown that safety is the focus of aborigines' concerns about block opening, so this study takes the possible losses caused by “potential” traffic accidents into consideration. The calculation formula is as follows [25]:

(19) $$\begin{array}{c} \min ARc=\sum_{ai\in Ai}0.0035\cdot l{}_{ai}^{0.6724}\cdot x_{ai}^{0.9679}\cdot Sc, \end{array}$$

where *ARc* is the loss cost of potential safety hazards, *Sc* represents the average cost of property damage per accident (including direct property damage and indirect property damage). It should be pointed out that the average period of each traffic accident is often long, so it is necessary to evenly allocate the cost to the same statistical time interval as other optimization objectives in actual calculation.

The above problems are transformed into a single-objective optimization model with the lowest cost, which is as follows.

(2) Decision variables: in this study, the decision variable of the upper-level planning model is the decision variable *yai* whether the road section is open or not:

(20) $$\begin{array}{c} yai=0,\;1ai\in Ai. \end{array}$$

In the formula, *yai*=0 means that road section *ai* is not open; *yai*=1 stands for section *ai* open in both directions.

(3) Constraints: the important purpose of opening blocks is to relieve the traffic pressure of urban main roads, but the traffic conditions inside blocks cannot be ignored, so the saturation of internal sections after opening blocks should be within the limit of maximum expected saturation.

(21) $$\begin{array}{c} Sai\leq \bar{S}ai\;ai\in Ai, \end{array}$$

where *Sai* is the saturation of the road section inside the block and $\bar{S}ai$ is the maximum expected saturation.

### 4.3. Experimental Comparison

Referring to the average block size of cities in China, the longest horizontal length of the block is set to 2.1 km and the longest longitudinal length is set to 1.8 km. Its external road network includes 34 intersection nodes, 38 two-way trunk roads, 26 two-way secondary trunk roads, and 11 urban branch roads. The interior of the block includes 9 intersections and 42 two-way branch roads. Taking Chengdu as an example, based on the actual data of the city, the parameters such as traffic capacity, driving speed, and travel demand of the example road section are set as follows: the single-side traffic capacity of the urban main roads in this area is 2200 Veh/h, and the speed is 40 km/h; the single-side traffic capacity of the secondary trunk road is 1800 Veh/h and the speed is 30 km/h, while the single-side traffic capacity of the branch road is 800 Veh/h and the speed is 30 km/h.

Suppose: when the traveler has low inertia decision, *φ*=0.2, *τ*   =   0.8; when the traveler has a low inertia decision, *φ*=0.35, *τ*   =   0.65; when the traveler has moderate inertia decision, *φ*=0.5, *τ*   =   0.5; when the traveler has high inertia decision, *φ*=0.65, *τ*   =   0.35; when the traveler has high inertia decision, *φ*=0.8, *τ*   =   0.2; and when the traveler is completely rational, *φ*=0, *τ*   =   1.

With the decrease of residents' travel decision inertia, the effect of opening blocks on relieving traffic pressure in urban sections is obviously improved. For example, although the travel cost inside the block becomes higher, the travel cost outside the block becomes lower, and the total system cost also becomes lower; the total travel time of the road outside the block decreased from 106,848 min to 101,116 min, a decrease of 5.36%. The results are shown in Figures 3 and 4.

In addition, after the opening of the block, the travel time of residents in the block is on the rise as a whole, and external vehicles can enter the inner lane of the block, which affects daily travel to some extent. As a result, the traffic road exhaust emissions and potential safety hazards in the block also show a positive growth trend. Among them, the exhaust emissions inside the block increased by about 3.7 times, and the value of potential safety hazards increased by about 3.6 times. The results are shown in Figure 5.

With the opening of the block roads, the average travel time of urban residents showed a downward trend, with an overall average decline time of about 33 min and a decrease of about 12.09%. Travel conditions have improved. The results are shown in Figure 6.

The result of these data is that when the traveler's decision inertia is high, the traveler is unwilling to transfer from the current choice to the better path in the block; however, when the traveler's decision inertia is low, the inner branch road of the block can be effectively utilized. Therefore, when implementing the block opening policy, the travel decision inertia of travelers can be reduced through reasonable information induction.

### 4.4. Optimization Results

By referring to other relevant professional contributions and simulation verification in this study, it is assumed that the tolerance coefficient *φ*=0.5, travel preference selection coefficient *τ*=0.5, maximum acceptable indifference threshold *ε*_max_^*w*^=0.25, traveler's travel time value *λ*=0.25, automobile unit operating cost $b_{a}=1\text{ yuan}/\text{km}\left(v=40\;\text{km}/\text{h}\right)-b\pm \sqrt{b^{2}-4ac}/2a$, *b*_*a*_=1.2(yuan/km)/(*v*=30 km/h)=30 km/h, environmental pollution loss cost *Q*_*c*_=0.1 yuan/g, and single accident loss cost *S*_*c*_=20亓/h, ${\bar{S}}_{a_{i}}=0.9$ of urban travelers in the system. Compared with before and after the optimization of the block road network, the total cost of the system changed to 113,820 yuan, a decrease of 2.63%. The travel time of the external section of the block road network decreased significantly, from 115,871 min to 103,674 min, a decrease of 10.53%. The average saturation of urban main roads decreased from 0.92 before opening to 0.87, a decrease of 6.23%, and the average saturation of secondary roads decreased from 0.84 to 0.74, a decrease of 11.56%. The congestion of the road network outside the block was obviously improved. However, some changes have taken place in the inner travel of the block. First, the travel time has increased from the initial 2125 min to 9264 min, and the average saturation of the road section has increased from the initial 0.14 to 0.58, which is still in a basically unblocked state. In addition, the emission of automobile exhaust pollution in the block increased by 1611 g/h, and the number of potential traffic accidents increased by 4.67/year, all of which may affect the daily life of residents.

## 5. Conclusion

In this study, the historical blocks are roughly divided into three modules for research, which are residential communities, cultural tourism areas, and traffic routes. The complete information game model is used to analyze the imbalance between property and residents. Adopt the AHP fuzzy evaluation method to detect the current life happiness coefficient of urban residents and collect residents' opinions and suggestions for the future planning of historical blocks. The bilevel programming model is used to solve the block road network optimization scheme, and the effectiveness of the optimization results is tested. The following conclusions are drawn:

1. Residents have high expectations for the safety and convenience of the future community, so we should focus on the research of future block planning from these two angles
2. Because the aging trend of today's social situation is getting worse and even more serious in the future, it is necessary to increase the community residents' service health platform. It is required to provide physical examination services or medical services for a certain period of time. At the same time, some health monitoring instruments can be installed, such as the pulse test, blood sugar test, and body fat measurement, which can provide residents with physical fitness tests free of charge at any time.
3. The commercialization of cultural tourism blocks is serious, the cultural atmosphere is not strong, and the main functions are not prominent. Therefore, it is of considerable practical significance to partition functional areas. The functions are divided into cultural area, retail sales of goods, specialty sales, and creative retail. At the same time, these four areas are connected by using Internet of Things technology to achieve the purpose of information sharing, real-time monitoring, and timely handling of emergencies.
4. Opening the entrance and exit of the block will help relieve the pressure on the main road, but it will also have a certain impact on the daily life of residents. The overall travel time of the block will decrease, but the travel time within the block, the incidence of safety accidents, and the emission of automobile pollution will increase. The decision inertia of urban travelers, the internal demand of blocks, and the demand of urban travel will also affect the opening effect of blocks. When the travel demand within the block is low (the average saturation of the internal road network is less than 0.6 under the condition of not opening the block) and the urban transit travel demand is high (the average saturation of the external road network is greater than 0.72 and less than 1.07), the open block can effectively alleviate the congestion of the external road network without obvious impact on the internal road network of the block. The higher the decision inertia of travelers, the higher the internal and external travel demand that the open block policy can cope with, that is, the stronger the adaptability of the policy.

## Figures and Tables

**Figure 1:** Weight relation diagram of primary and secondary levels.

**Figure 2:** Functional partition.

**Figure 3:** Travel cost change.

**Figure 4:** Total travel time of road network sections.

**Figure 5:** Exhaust emissions and potential safety hazards.

**Figure 6:** Average travel time of travelers.

**Table 1:** Game between owners and property management companies.

		Residents, *N*1	
		Regular payment	Deferred payment
Property company, *N*2	Quality service	*M*+*E*1 − *C*1, *R*1	*M* − *C*1, *R*1+*E*1
	Low-quality service	*M*+*E*1 − *C*2, *R*2	*M* − *C*2, *R*2+*E*2

**Table 2:** Scores of each evaluation index.

Criterion level	Score	Index level	Score
Safety	9.1	Community security	8.7
		Personal safety of residents	8.9
		Residents' property safety	8.1

Convenience	8.5	Convenience of residents' life	7.5
		Degree of difficulty resolution	6.1

Reliability	7.6	Property safety for residents	8.3
		Property guarantees for residents' living services	7.8

Rapidity	6.3	Speed of life service provided by property	6.5
		The speed of solving the difficulties of residents by property	7.1

Economy	7.1	Proportion of residents' contributions	7.3
		Quality of property services	8.6

Comforts	8.6	Community greening environment	7.8
		Community safety environment	8.8
		Residents' happiness index	7.1
		Home care	8.7

**Table 3:** “Security” weight set.

*B*_1_	*C*_1_	*C*_2_	*C*_3_	*K*_*i*_
*C*_1_	1	0.3	0.1135	0.0748
*C*_2_	5	1	1/3	0.2563
*C*_3_	9	3	1	0.6754

**Table 4:** Evaluation weight of residents' satisfaction with open community.

Weight value	Safety 0.4236	Convenience 0.0831	Reliability 0.1349	Rapidity 0.0283	Economy 0.2496	Comfort 0.0325	Total weight value of C layer sorting	Importance ranking
Community security	0.0597	0	0	0	0	0	0.2894	2
Personal safety of residents	0.3214	0	0	0	0	0	0.3657	1
Residents' property safety	0.6950	0	0	0	0	0	0.1357	4
Convenience of residents' life	0	0.7241	0	0	0	0	0.2647	3
Degree of difficulty resolution	0	0.1883	0	0	0	0	0.0134	15
Property security for residents	0	0	0.0532	0	0	0	0.0754	6
Residents' living service guarantee	0	0	0.0401	0	0	0	0.0271	9
Life service speed provided by property	0	0	0	0.2374	0	0	0.0134	14
The speed of solving the difficulties of residents by property	0	0	0	0.4879	0	0	0.0548	8
Residents' contribution ratio	0	0	0	0	0.1130	0	0.0225	1
Property service quality	0	0	0	0	0.2713	0	0.0628	7
Community greening environment	0	0	0	0	0	0.5328	0.0040	12

**Table 5:** Comparison table of speed correction factor values of small vehicles.

Pollutant	Velocity interval (km/h)				
	<20	20–30	30–40	40–80	>80
CO	1.69	1.26	0.79	0.39	0.62
HC	1.68	1.25	0.78	0.32	0.59
NO_*x*_	1.38	1.13	0.90	0.86	0.96

## Data Availability

The data used to support the findings of this study are available from the corresponding author upon request.
